The article "Classification and Reconstruction of Biomedical Signals Based on Convolutional Neural Network" was published in 2022. Journal: Comput Intell Neurosci.

# Classification and Reconstruction of Biomedical Signals Based on Convolutional Neural Network

**DOI:** 10.1155/2022/6548811

**Published:** 2022-07-21

**Authors:** Zijiang Zhu, Hang Chen, Song Xie, Yi Hu, Jing Chang

**Affiliations:** ^1^School of Computer Science, South China Business College, Guangdong University of Foreign Studies, Guangzhou 510545, Guangdong, China; ^2^Institute of Intelligent Information Processing, South China Business College, Guangdong University of Foreign Studies, Guangzhou 510545, Guangdong, China; ^3^Information Engineering School, Guangzhou Vocational College of Technology & Business, Guangzhou 511442, Guangdong, China

## Abstract

The efficient biological signal processing method can effectively improve the efficiency of researchers to explore the work of life mechanism, so as to better reveal the relationship between physiological structure and function, thus promoting the generation of major biological discoveries; high-precision medical signal analysis strategy can, to a certain extent, share the pressure of doctors' clinical diagnosis and assist them to formulate more favorable plans for disease prevention and treatment, so as to alleviate patients' physical and mental pain and improve the overall health level of the society. This article in biomedical signal is very representative of the two types of signals: mammary gland molybdenum target X-ray image (mammography) and the EEG signal as the research object, combined with the deep learning field of CNN; the most representative model is two kinds of biomedical signal classification, and reconstruction methods conducted a series of research: (1) a new classification method of breast masses based on multi-layer CNN is proposed. The method includes a CNN feature representation network for breast masses and a feature decision mechanism that simulates the physician's diagnosis process. By comparing with the objective classification accuracy of other methods for the identification of benign and malignant breast masses, the method achieved the highest classification accuracy of 97.0% under different values of *c* and gamma, which further verified the effectiveness of the proposed method in the identification of breast masses based on molybdenum target X-ray images. (2) An EEG signal classification method based on spatiotemporal fusion CNN is proposed. This method includes a multi-channel input classification network focusing on spatial information of EEG signals, a single-channel input classification network focusing on temporal information of EEG signals, and a spatial-temporal fusion strategy. Through comparative experiments on EEG signal classification tasks, the effectiveness of the proposed method was verified from the aspects of objective classification accuracy, number of model parameters, and subjective evaluation of CNN feature representation validity. It can be seen that the method proposed in this paper not only has high accuracy, but also can be well applied to the classification and reconstruction of biomedical signals.

## 1. Introduction

Biomedical signals can be a class of signals originating from a biological system, and these signals usually contain information related to the physiological and structural state of the biological system. There are many kinds of biomedical signals, and their main characteristics are weak signals and large randomness. With the rapid development of digital medical technology and biological technology, scholars in related fields have a growing demand for processing and analyzing biomedical data. Relying solely on researchers or doctors to manually record, collate, and query related research data and clinical information, traditional biomedical information processing methods can no longer meet the growing demand for large-scale, quantitative biomedical information analysis. Committed to the practice in the fields of biology and clinical medicine, the research on biomedical informatics, which comprehensively studies and applies information science, computer science, cognitive science, and brain-machine interaction, is gradually emerging. Biomedical signals are the most direct description of the state of living things that can be collected by instruments and equipment. It is an important research object in biology, informatics, medicine, and so on. With the rapid development of biomedical-related disciplines, researchers and medical workers have an increasingly strong demand for such signal processing and analysis technologies. Efficient biological signal processing methods can effectively improve the efficiency of researchers to explore the work of life mechanisms, so as to better reveal the relationship between physiological structure and function, thus promoting the production of major biological discoveries. High-precision medical signal analysis strategy can, to a certain extent, share the pressure of doctors' clinical diagnosis and assist them to formulate more favorable plans for disease prevention and treatment, so as to alleviate patients' physical and mental pain and improve the overall health level of the society. Traditional signal analysis methods have been difficult to meet the increasing demands of biomedical signal processing, and the use of advanced machine learning technology to effectively model and analyze the involved problems has become a research hotspot in this field. Breast cancer is one of the most common female malignant tumors, accounting for 24.2% of the total malignant tumors. The incidence of the population varies from region to region. The more developed the region, the higher the incidence of breast cancer.

As one of the new effective signal processing tools, neural network has the advantage that other signal processing tools cannot solve technical problems [1]. It is widely used in many fields, especially in biomedical engineering [2]. Deep learning is a machine learning method that uses multi-layer neural network to obtain the feature representation of data and then use the feature representation for data analysis. As the most concerned research direction in the field of machine learning, deep learning is leading a new wave of artificial intelligence research. With its strong nonlinear feature representation ability, in recent years, the convolutional neural network has become the most widely applied deep learning model with the best comprehensive effect and has made a series of unprecedented breakthroughs in many tasks represented by pattern recognition [3].

Inspired by the success of convolutional neural network in other fields and combining with the characteristics of specific biomedical signals, this paper proposed several classification and reconstruction methods of biomedical signals based on convolutional neural network, taking mammography images and EEG signals as research objects [4, 5]. The main innovations of this paper are as follows:

1. In the classification task of breast lumps based on molybdenum target X-ray, the design can effectively describe the visual characteristics of breast lumps, and it is the key to complete high-precision auxiliary diagnosis to easily distinguish the visual characteristics of benign and malignant lumps in the feature space. In this paper, a classification method of benign and malignant breast lumps based on the characteristic representation of convolutional neural network is proposed [6]. In this method, a network was constructed to represent the visual features of the tumor image, and the network was trained based on the natural image and the breast image. Then, by referring to the actual diagnosis experience of doctors, the network was used to obtain the description of visual features at different levels suitable for the classification of breast lumps. Finally, a decision mechanism for the characteristics of breast lumps was proposed to determine the benign and malignant breast lumps. The experimental results show that this algorithm can effectively describe the features of convolutional neural network and realize the classification of benign and malignant breast lumps with high accuracy. (2) In the computer-aided diagnosis of breast diseases, atypical samples with insignificant visual characteristics are often encountered [7]. In the traditional manual visual feature space and convolutional neural network feature space, this type of sample cannot be effectively described. It is an effective way to solve this problem to map the samples that cannot be effectively described in the original feature space to the easily distinguished feature space through the feature space transformation operation. Therefore, an improved convolutional neural network model based on large interval measurement learning is proposed for the classification of breast lumps. To be specific, firstly, the mapping relationship from the original convolutional neural network feature space to the new feature space is learned by introducing the large interval measure learning loss function. From the mapping relationship, the features of breast masses with tighter intra-class distribution and more discrete inter-class distribution were obtained. In addition, network training improvement strategy focusing on difficult cases is proposed by providing new error samples to the network continuously. The experimental results show that the learning layer of the algorithm can improve the discrimination of features and the accuracy of network classification, and the improved network training strategy can further improve the performance of the network in the task of differentiating benign and malignant breast masses. (3) In the task of neural decoding based on EEG signals, classification of EEG signals caused by different types of stimuli is one of the basic tasks in this field [8]. EEG signal contains abundant spatiotemporal characteristics, and the traditional EEG signal feature description method can only represent one of these characteristics, failing to provide a more effective feature representation basis for subsequent classification tasks. To solve the above problems, this paper proposes a classification method of EEG signals based on spatiotemporal fusion convolutional neural network. Specifically, firstly, different methods of generating EEG were used to generate EEG focusing on spatial information and temporal information. Then, the convolutional neural network which can feature two different activation graphs is designed and trained, respectively, to obtain the convolutional neural network feature representation of EEG signals. Finally, two fusion methods of feature splicing and feature selection were used to classify EEG signals. Experimental results show that the feature representation part of this algorithm can obtain the EEG feature representation with strong discriminability, and the subsequent spatial-temporal fusion strategy can further improve the classification accuracy of EEG signals. (4) Visual stimulus reconstruction based on EEG signals is another typical neural decoding task based on high-precision EEG signal classification [9, 10]. This task is usually composed of two stages: high-precision EEG signature representation and classification, and visual stimulus generation. In the traditional visual stimulus reconstruction method based on cognitive spatial EEG characteristics, limited by the limit of human cognitive level and the error of neural signal acquisition process, it is difficult to achieve significant improvement in classification accuracy and representation efficiency. Inspired by the results of the current convolutional neural network in visual tasks beyond human performance, this paper proposes a visual feature-guided classification method for EEG signals. By mapping the representation of EEG signals to visual space, this method can classify EEG signals with higher accuracy. Then, based on the EEG representation guided by visual features, this paper proposes an improved generation antagonism network model for generating visual stimuli. The experimental results of EEG signal classification and visual stimulus generation show that this algorithm can effectively improve the accuracy of EEG signal classification and the quality of visual stimulus reconstruction results.

## 2. Proposed Method

### 2.1. Biomedical Informatics

Neural network is adaptive, which refers to the ability of a system to change its performance to adapt to changes in the environment. When the environment changes, it is equivalent to inputting new training samples to the neural network. The network can automatically adjust the structural parameters and change the mapping relationship, so as to generate the corresponding expected output for the specific input. Therefore, the neural network has stronger adaptability than the expert system using the fixed reasoning method and is closer to the operation law of the human brain. With the rapid development of digital medical technology and biological technology, scholars in related fields have a growing demand for processing and analyzing biomedical data [11]. Relying solely on researchers or doctors to manually record, collate, and query related research data and clinical information, traditional biomedical information processing methods can no longer meet the growing demand for large-scale, quantitative biomedical information analysis. Committed to the practice in the fields of biology and clinical medicine, biomedical informatics research on information science, computer science, cognitive science, and brain-machine interaction has gradually emerged [12]. The purpose and task of biomedical signal processing are to determine the state of the system (normal, pathological) from the characteristics of the analysis signal, so as to achieve the purpose of making accurate medical decisions.

Medical image processing institutions around the world have rapidly entered the field and applied CNN and other deep learning methods to various medical image analyses. As a new and interdisciplinary research field, biomedical informatics and traditional biology, computer science and clinical medicine research are interdependent and collaborative. Biology, clinical medicine, and computer science, respectively, provide theoretical support, practical support, and technical support for biomedical informatics research [13, 14]. At the same time, biomedical informatics also provides effective methods and theoretical reference for the communication and interdisciplinary research among other disciplines. It is an important bridge and link for carrying out interdisciplinary research in related fields, and can well promote the comprehensive and coordinated development of various disciplines. The relationship between biomedical informatics and other disciplines is shown in Figure 1.

According to different research objects and application fields, the main research directions of biomedical informatics include the following:

1. Bioinformatics is a discipline that explores objective laws existing in complex biological data according to biological research methods and principles through advanced computer science and technology [15]. The core problem is to design efficient software or develop more advanced data processing methods for how to organize and understand biological data more effectively [16]. At present, the research work of bioinformatics mainly focuses on gene sequence analysis, biodiversity measurement, protein structure prediction, and protein and gene expression analysis [17]. Gene sequence analysis, for example, phage Φ - X174, is the first measured complete genome sequences of an organism. Since then, gene sequences of thousands of organisms have been measured gradually, providing new ideas for the diagnosis and treatment of human genetic diseases and the selection and breeding of superior crop varieties. With the increasing complexity of gene sequences, it is impossible to compare and analyze gene sequences by hand. To BLAST (Basic Local Alignment Search Tool) as the representative of analysis software has gradually become the backbone of gene sequence analysis. Today, analysis tools such as BLAST help scientists around the world analyze more than 190 billion nucleotides a day, greatly increasing the efficiency of gene sequencing [18]. Convolutional neural network (CNN) is mainly used in the field of image recognition. It refers to a class of networks, rather than a certain kind of network, which includes many networks with different structures. Different network structures usually behave differently.
2. Pharmacoinformatics is a multidisciplinary discipline of computer science, life science, mathematics, and other theoretical methods, aiming at more scientific and reasonable drug design and development [19, 20]. As a relatively late branch of biomedical informatics, the main research object of pharmaceutical informatics is the information directly or indirectly related to drugs represented by the action mechanism of drugs, adverse drug reactions, and drug interactions. The focus of clinical pharmacy research is to use the professional knowledge of pharmacy to serve patients, and its purpose is to improve the quality and level of medical care. Pharmacy information plays an important role in the monitoring of drug concentration in the treatment clinic and obtaining relevant pharmacokinetic parameters as well as the relationship between drugs and disease, drug resistance, and patient health information that are indirectly related to drugs. In drug design, for example, supervised machine learning method (supervised machine learning) was used to explore drug structure and its effect, and the relationship between and according to the structure of new drug efficacy of prediction guide the design and r&d of new drugs. The basic method of medical inspection image processing is digital filtering: because in the process of image acquisition, it will inevitably bring a lot of random noise, and various digital filtering on the digitized image signal will greatly improve the quality of the image quality.
3. Medical Image Analysis. The research object of medical image analysis is a variety of biomedical images, and its main research contents include the collection, storage, compression, registration, analysis, and other technologies of medical images [21]. In recent years, with the development of computer-aided diagnosis technology, image enhancement, super-resolution, lesion detection, segmentation, and 3d reconstruction based on machine learning methods have become the focus of research in the field of medical image graphics [22]. Taking the diagnosis of pneumonia based on chest X-ray as an example, the network is trained with a large number of labeled lung X-ray images. The current advanced deep convolutional neural network model can achieve or even exceed the performance of radiologists in such tasks [23].

### 2.2. Biomedical Signals

As the main carrier of biomedical informatics research, biomedical signal is an important research object in biomedical informatics [24]. Based on whether the signals collected are directly from the spontaneous physiological activities of human beings or other living organisms, common biomedical signals can be classified as follows:

1. Spontaneous signals. The signals are spontaneously generated during the physiological activities of human beings or other living bodies, such as electrophysiological signals such as electroencephalogram, electrocardiogram, electroencephalogram, and nonelectrophysiological signals such as body weight and respiration [25–27]. Among them, electrophysiological signals can provide abundant data for human vision, psychology, neuroscience, and other research directions; nonelectrophysiological signals can provide early support and basic guarantee for scientific research and clinical diagnosis and treatment of disease prevention and preliminary diagnosis and daily observation of disease changes.
2. Passive signal. Another kind of biomedical signal is a variety of passive signals collected by external instruments upon the human body, including a variety of common medical imaging methods: such as MRI, computed tomography, ultrasound, and positron emission tomography [28, 29]. According to the difference in physical characteristics of the imaging site, different passive biomedical signals have their advantages in related researches. For example, X-ray-based CT images have high contrast and spatial resolution when imaging dense tissues. The ultrasonic imaging method has no harm to human body and is suitable for the daily examination of pregnant women and other sensitive people. MRI equipment not only does not have the harm of ionizing radiation, but also can provide high resolution, which has significant advantages in the examination of brain and spinal cord diseases and angiography. Through quantitative and dynamic detection of changes in cell metabolites or drugs, PET imaging has become the best method to diagnose and guide the treatment of various malignant tumors, coronary heart disease, and brain diseases [30, 31]. The acquisition objects of biomedical signals are generally human or other complex living bodies, and the acquisition conditions include the living body's internal environment and external environment with individual differences.

### 2.3. Classification of Breast Masses Based on CNN Features

Breast magnetic resonance imaging technology has the characteristics of excellent soft tissue resolution and no radiation and has unique advantages in breast examination. Especially with the development and application of special breast coils and rapid imaging sequences, the quality and level of breast magnetic resonance images have been greatly improved. Breast cancer is of the highest incidence of malignant tumors in women all over the world, it is often considered the common diseases of the population in developed countries, but nearly 50% of breast cancer cases and 58% of deaths occur in less developed countries. As shown in Table 1, according to the authoritative World Health Organization (WHO) statistics, breast cancer, which accounts for 29% of the total number of diagnosed cancers in women, is one of the main causes of cancer-related deaths in women, and it poses a great threat to women's health. Although the incidence of breast cancer in Asian women is slightly lower than that in white women, the incidence of breast cancer in Chinese women has been on the rise in recent years. Adenocarcinoma is a serious threat to women's health, and the global incidence of breast cancer has been on the rise since the late 1970s. According to relevant statistics, the global incidence of breast cancer is 24.2%, of which the majority are in developing countries. At the same time, due to the lack of sufficient attention to breast cancer, prevention propaganda is relatively not in place, the survival rate of female breast cancer patients in China is far lower than that in Western countries, and the age of onset of female breast cancer is far lower than the average level in Western countries. Early detection of breast cancer greatly increases the likelihood of successful treatment plan, and a computer-aided diagnosis is mainly for early detection of breast cancer, to achieve more rapidly and accurately for the purpose of the breast cancer diagnosis, effectively improve the 5-year survival rate for patients with breast cancer and 10-year survival rate, and greatly reduce the disease to patients and patients' families suffering physical and mental damage. At present, the early diagnosis of breast cancer mainly includes doctor's touch, tissue biopsy, and imaging examination. Among them, the doctor's touch test is more dependent on the doctor's experience and is more likely to be affected by the individual physical characteristics of the patient. It is difficult to find early and small breast lumps, and is usually only used as an auxiliary means to cooperate with other types of examination. However, biopsy usually involves puncturing the patient's breast, which can cause greater physiological pain to the patient and is usually only used as pathological analysis after the removal of suspected malignant tissue.

With the continuous development of medical imaging technology, image-based breast examination has become the most widely used method for early diagnosis of breast cancer. Mammography, CT, ultrasound, and MRI are the most common imaging methods of breast tissue [32]. Among them, breast ultrasound does not produce any ionizing radiation, but its imaging quality is relatively poor. It is usually used in sensitive groups such as pregnant women or as an auxiliary strategy for other examination means. The CT imaging effect of breast is good, but the relative radiation dose is large, which is not suitable for regular examination and sensitive population. The quality of breast MRI imaging is high and can be enhanced by contrast agent, but the cost is high, and the hardware required for examination is not available in areas with relatively poor medical environment, which is not conducive to long-term and large-scale application. Compared with other common examination methods mentioned above, mammography has the advantages of low examination cost, relatively small radiation dose and high definition. Image-based breast examination has become the most widely used method for early diagnosis of breast cancer. Mammography, CT, ultrasound, and MRI are the most common imaging methods for breast tissue. Among them, breast ultrasound does not produce any ionizing radiation, but its imaging quality is relatively poor. It is usually used in sensitive groups such as pregnant women or as an auxiliary strategy for other examination means. On the basis of the classification method of breast lumps based on the classical manual visual feature combining classifier, and inspired by the successful application of CNN model in many medical image analysis tasks mentioned above, the classification method of breast lumps based on CNN feature representation was proposed. The method consists of CNN feature representation network and a series of CNN feature decision mechanism.

#### 2.3.1. CNN Feature Representation Network of Breast Mass

A convolutional neural network of *L* layers, with input of *x*_1_,  *x*_2_,…, *x*_*L*_ for each layer and connection weight of *W*_1_, *W*_2_,…, *W*_*L*_ for each layer, is structurally equivalent to that shown in Figure 2, with *L* filters *f*_1_, *f*_2_,…, *f*_*L*_ directed acyclic graph.

Inspired by the classic LeNet, AlexNet CNN network structure, this paper introduces the characteristics of breast masses. The CNN network is mainly composed of a series of convolution and connection layers. This paper divides breast features into five convolutional modules, 3 fully connected layers, and Softmax loss function, where each convolutional layer contains a pooling layer and an activation layer or a convolutional layer and an activation layer. Convolution operation is considered to be able to simulate directional selection neurons in the primary visual cortex of human brain. Convolution module is an indispensable part of CNN model. Assuming that the input of the convolutional layer is the tensor *x* of the K channel, the convolutional layer is composed of K multi-channel convolutional kernel *f* with bias *b*. *H*, *W*, and *D*, respectively, represent the height, width, and channel number of input *x*; *H*′, *W*′, and *D* represent the height, width, and number of channels of the convolution kernel, respectively; *H*″, *W*″, and *K*, respectively, represent the height, width, and channel number of the output *y*; *D*, *d*′, and *d*″, respectively, represent channel indexes of convolution kernel *f*, input *x*, and output *y*. Then, the operation of the convolutional layer is

(1) $$\begin{array}{c} y_{i^{\prime \prime }j^{\prime \prime }d^{\prime \prime }}=b_{d^{\prime \prime }}+\sum_{i^{\prime }=1}^{H^{\prime }}\sum_{j;=1}^{W^{\prime }}\sum_{d^{\prime }=1}^{D}f_{i^{\prime \prime }j^{\prime \prime }d^{\prime \prime }}\times x_{i^{\prime \prime }+i^{\prime }-1,j^{\prime \prime }+j^{\prime }-1,d^{\prime },d^{\prime \prime }}, \end{array}$$

where, *I*′, *J*′, respectively, represent the high and wide position index of convolution kernel; *I*′, *J*′, respectively, represent the high and wide position index of output *y*. In CNN model, the maximum value pooling strategy is used for the pooling operation. The maximum value pooling method selects and calculates the maximum response value of each characteristic graph within the block range of *H*′ × *W*′. If *x* is the input of the maximum pooling layer and *Y* is the output of the layer, the operation of the maximum pooling layer can be expressed as follows:

(2) $$\begin{array}{c} y_{i^{\prime \prime }j^{\prime \prime }d^{\prime \prime }}=\underset{1\leq i^{\prime }\leq H^{\prime },1\leq j^{\prime }\leq W^{\prime }}{\max}x_{i^{\prime \prime }+i^{\prime }-1,j^{\prime \prime }+j^{\prime }-1,d}, \end{array}$$

where *I*″ and *j*″ represent the high and wide position indexes of input *x* and output *y*, *I*′ and *j*′, respectively, represent the high and wide position indexes of *H*′ × *W*′ range, and *d* represents the feature graph channel indexes of input and output. The modified linear element is selected as the activation function in the CNN model. This activation function has the characteristics of unilateral inhibition, relatively wide excitation boundary, and sparse activation, which is proved to be more similar to the working principle of human cortical neurons. Similarly, if the input of the activation function is *x* and the output is *y*, then the operation of this layer is

(3) $$\begin{array}{c} y_{ijd}=\max\left\{0,x_{ijd}\right\}, \end{array}$$

where *I*, *j*, and *d* represent the height, width, and channel indexes of input and output, respectively. After a series of convolution, pooling, and activation operations, in the CNN model, the image feature representation has been transformed from feature graph to high-dimensional feature vector. The operation of full connection in the two adjacent full connection layers is completed by matrix multiplication. Suppose the input of the full connection layer is *x* and the output is *y*, then

(4) $$\begin{array}{c} y=C_{x}+b, \end{array}$$

where *C* is the connection weight of the full connection layer and *b* is the offset of the full connection layer. The main function of the all-connected layer is to transform the representation of feature vectors in different feature spaces. In addition, referring to the representative work of CNN model training strategy, we added batch normalization operation after the convolution operation of Conv1 of the first volume layer and Conv5 of the fifth convolutional layer of the network. Suppose that the data before the batch normalization are *x*, the processed data are *y*, *M* is the connection weight of the layer, *b* is offset, *M* ∈ *R*^*D*^, *b* ∈ *R*^*D*^, *x*, *y* ∈ *R*^*H*×*W*×*D*×*T*^, *H* stands for the height of the feature graph, *W* stands for the width of the feature graph, *D* stands for the number of channels of the feature graph, and *T* stands for the number of image input into the network of the same batch during the training process, then the batch normalization operation can be expressed as

(5) $$\begin{array}{c} y_{ijdt}=M_{d}\frac{x_{ijdt}-}{\sqrt{\sigma 2d+\varepsilon }}b_{d},\\ \mu_{d}=\frac{1}{HWT}\sum_{i=1}^{H}\sum_{j=1}^{W}\sum_{t=1}^{T}x_{ijdt},\\ \sigma_{d}^{2}=\frac{1}{HWT}\sum_{i=1}^{H}\sum_{j=1}^{W}\sum_{t=1}^{T}{\left(x_{ijdt}-\mu d\right)}^{2}. \end{array}$$

### 2.4. Visual Stimulus Reconstruction Method Based on EEG and Generation against CNN

If we assume that EEG signals and their corresponding representations exist in the cognitive space, and visual stimuli and their corresponding representations exist in the visual space, the existing neural decoding methods based on EEG signals can be summarized into two stages: the classification stage of EEG signals in the cognitive space; the EEG signal characteristics of cognitive space are used to guide the classification and generation of visual stimuli in visual space. The premise that this kind of method can achieve higher precision decoding results is that the human brain performs better in related tasks than the machine learning method based on the representation of computer vision features. However, with the continuous progress of computer visual feature representation methods based on various deep learning models, the performance of deep learning structures represented by CNN in visual feature representation and classification tasks has surpassed the level of human beings. As a result, the ability to decode EEG signals in cognitive space alone, or to use EEG signals to guide the decoding of visual stimuli, is limited by the upper limit of the brain's ability to perform related visual tasks. In order to obtain the results of neural decoding with higher accuracy, we proposed a visual stimulus reconstruction method guided by CNN visual features and based on EEG signals. The method can be divided into two stages: CNN visual feature representation-guided EEG signal classification and generation-based visual stimulus generation against CNN.

## 3. Experiments

### 3.1. Breast Mass Image Data

#### 3.1.1. Data Source

The breast mass data used in this study came from DDSM, the most widely used and largest mammography data set, which was compiled and published by the University of South Florida and contains classification labels for benign and malignant breast lumps and pixel-level accurate labeling information for lesion areas. The data set parameters and content settings used in this paper are consistent with previous studies, and there are 300 images of benign tumor and 300 images of malignant tumor in the data set. Breast mass data were divided into training set, validation set, and test set according to the proportion of 50%, 25%, and 25%, with the same number of benign and malignant lumps in each set.

#### 3.1.2. Objective Evaluation

In order to objectively evaluate the effectiveness of our method, we chose the average classification accuracy (the average result of 200 random partitions) of the data set of multiple random partitions as the objective evaluation standard by referring to previous relevant research literature. In terms of the image data of breast lumps based on in this chapter, we made a comparison with the current mainstream classification methods of breast lumps, including (1) MLP: classification method of benign and malignant breast lumps based on the grade of breast disease, patient age, other characteristics, and multi-layer perceptron; (2) FA: benign and malignant tumor classification method/based on local texture characteristics and fractal analysis (FA); (3) GLBI: the classification method of benign and malignant breast tumors based on grayscale characteristics and grade of breast tumors; (4) SCN: benign and malignant tumor classification method based on soft clustering network; (5) LFM: lump classification method based on hidden feature mining and visual word bag model; and (6) CNN: the tumor classification method based on CNN feature representation proposed in this paper.

### 3.2. Experimental Data of Visual Stimulus Reconstruction Method Based on EEG and Generation against CNN

The EEG data used in this study were derived from the event-related potential experiment induced by visual stimuli. A total of 6 subjects participated in the data acquisition experiment. Physical function of 6 subjects was normal. Each subject was required to view images of 40 categories with 50 samples in each category, and the total display time of each category was 25 seconds (i.e., 0.5 seconds for each image). A 10-second display of a pure black background between images of different classes clears the mind of the previous category. The EEG acquisition equipment used in the experiment was 128 lead EEG signal receiving and amplifier produced by Brain Products of Germany. The collected EEG signals were processed by a second-order Butterworth bandpass filter with a frequency range of 14–70 hz to obtain EEG signals containing the range of human cognitive information. The corresponding 40 visual stimulus images were from the ImageNet image data set.

### 3.3. GAN Network Structure and Training Data

The GAN model proposed in this paper for generating visual stimuli consists of a discriminant network *D*, a generating network *G*, and a feature representation network *R* shared by two parameters. Network *D* is the convolution network, and its main network parameters are shown in Table 2, where Conv stands for convolution operation, BN stands for batch normalization, and ReLU stands for activation function. The generated network *G* is the deconvolution network, where Deconv stands for deconvolution operation, BN stands for batch normalization, and ReLU stands for activation function. *R* network is pretrained full convolution network FCN−8s. The training of GAN adopts Adam method, the learning rate is set to 0.0002, and the sample number of a single input network is 16.

## 4. Discussion

### 4.1. Verification and Analysis of Breast Image Data Set

This section validates the proposed method on the most widely used breast image data set and analyzes the proposed method from two aspects of objective evaluation and subjective evaluation.

#### 4.1.1. Objective Evaluation and Analysis

The classification accuracy of the CNN feature representation method and the traditional manual visual feature method is shown in Figure 3.

It is easy to find from the statistical results of Figure 3: one is based on traditional manual method (MLP) which requires fusion of the visual identity of the gray scale, texture, and other different kinds of visual features, and this kind of feature fusion process parameter settings is relatively complex and needs to separate design or into other machine learning methods to complete the breast lump visual feature fusion operations. In addition, MLP and GLBI need to be considered in the inspection of visual features of patient age, because information from different modalities can achieve high-precision mass classification, but in the actual diagnosis and treatment process, there are usually only single-modality bump images. However, the needs of this multimodal information fusion method obviously cannot better meet the needs of actual diagnosis and treatment. However, the proposed method only uses the same CNN feature to represent the depth characteristics of different layers in the network and the simple decision-making mechanism can achieve the classification results of benign and malignant tumors with high accuracy. The average accuracy of the method proposed in this paper is above 85%, while the accuracy of the common method is only within 10%.

In the feature decision mechanism we proposed, SVM classifier is used to judge the feature representation of different layers. The commonly used SVM classifier forms are linear SVM and SVM based on radial basis function. SVM classifier based on RBF needs to adjust parameters *c* and gamma to obtain the best classification effect. We have 2^−14^, 2^−15^,…. In the range of 2^14^, 2^15^, parameters are selected for the performance of RBF-based SVM under the feature decision mechanism proposed by us. When *c* = 2^5^ and gamma = 2^−12^, the highest classification accuracy was 97.0%, which was only slightly higher than the performance of linear SVM (96.7%), which did not need parameter adjustment and had faster training speed. Therefore, considering the efficiency and accuracy of the algorithm, we chose linear SVM during the implementation of the feature decision mechanism. By further comparing and utilizing the proposed decision mechanism, the experimental results based on different convolutional neural network models are shown in Table 3.

In Table 3, we further compare the experimental results based on different convolutional neural network models using the proposed decision mechanism. It can be found that the network structure we used can achieve high-precision classification of breast masses under the condition of keeping the minimum number of parameters and occupying the minimum storage space. Its accuracy is only slightly lower than that of VGGNet, which has huge storage consumption and model parameters.

#### 4.1.2. Subjective Evaluation Analysis

We further introduced the feature vector distribution visualization method to evaluate the validity of CNN feature representation of breast tumors. We adopt the t-sne method, which is widely used in deep learning, for feature vector reduction and 2d display. This method by affine transformation in the high-dimensional space data points (eigenvectors) is mapped to a Gaussian distribution, at the same time in low-dimensional space with student's *t*, building and the corresponding data points of probability distribution, and by minimizing the distance between two probability distributions to complete mapping from high-dimensional feature space to low dimension space and achieve in low-dimensional space visualization of high-dimensional feature vector distribution. In the generated visual images, the easier it is for the sample points of different categories to be distinguished, the better it is proved that the feature is distinguishable and more effective for the classification task. We chose the gray-level feature of the original bump image, the middle-level CNN feature representation (Conv5) of the bump image, and the higher-level CNN feature representation (Fc7) of the bump image used in the discrimination mechanism for t-sne visualization, and the results are shown in Figure 4. In Figure 4, orange dot represents the benign tumors and blue point represents the malignant tumors. The visualization results of different layer features in the comparison graph show that the middle and top features of the network bump represented by CNN are much more distinguishable than the original massive data, and the features represented by CNN can effectively increase the difference between malignant tumor samples and benign tumors. The results also verify the validity of our proposed CNN feature representation network subjectively.

Based on the comparison between results of different layer visualization, we can draw the following. Network CNN characteristics of different layer can depict mass characteristics of different levels and high-level features tend to bump the overall characteristics of the middle and the underlying characteristics of mass containing more detailed information; this is related to the different degrees of diagnostic requirements for doctors to consider the visual features of breast lumps in actual clinical images.

### 4.2. Visual Stimulus Reconstruction Analysis Based on EEG and Generation against CNN

Vision is one of the most important human senses, which is mainly produced by the action of light stimulation on the human eye. And light is a visual stimulus, light is electromagnetic radiation with a certain frequency and wavelength, and in the vast electromagnetic radiation, visible light is only a narrow area, that is, the suitable stimulus for vision, and the suitable stimulus wavelength is 380∼780 nanometers. Light outside this range is invisible to the human eye. The visual reconstruction method proposed in this paper includes the classification of EEG signals and the generation of visual stimuli, so the analysis of the results is also carried out from the accuracy of EEG signal classification and the quality of visual stimulus generation results.

#### 4.2.1. Accuracy Analysis of EEG Classification

Classification accuracy was selected as the objective evaluation standard for EEG signal classification. The accuracy of the current mainstream EEG signal classification methods and the visual guided classification methods we proposed are shown in Figure 5.

By comparing the results in this figure, it can be found that the classification accuracy of the visual feature-guided classification method proposed by us is significantly improved compared with the classification method based on single cognitive space EEG signal (including CNN based on deep learning model, LSTM and LDA based on traditional machine learning method). Of the several visual signals used in this paper to guide classification, the feature representation provided by ResNet101 is most helpful in improving the accuracy of EEG signal classification, reaching the highest classification accuracy at present.

In addition, the t-sne feature visualization method adopted in previous sections of this paper was selected as the subjective evaluation standard for EEG classification tasks. In order to compare the difference between the visually guided EEG signal representation and the EEG signal representation in the traditional cognitive space, we chose the EEG signal representation obtained by the CNN method with the best performance in the cognitive space and the EEG signal representation after regression to the visual feature as the visual object. The visualization results are shown in Figure 6.

The dots of different colors in Figure 6 represent 40 types of visual stimulus image samples. The better the discrimination between different types of samples, the more suitable the characteristics are for EEG signal classification. The sample discrimination of different feature representation methods in the figure is consistent with the variation trend of classification accuracy of corresponding methods in Figure 5. The EEG feature representation guided by visual features is more compact within the class and more discrete between the classes, which makes the visual feature representation more conducive to the improvement of classification accuracy than the EEG feature representation in a single cognitive space.

In the EEG signal classification stage, the visual feature guidance strategy proposed in this paper can break through the limitation of the feature representation of EEG signals in a single cognitive space and effectively improve the accuracy of EEG signal classification by virtue of the powerful representation and discrimination ability of CNN visual features. In the visual stimulus generation stage, the EEG signal expression guided by visual features we adopted can provide effective guidance information for the generation of visual stimuli conforming to the EEG signal description. In addition, we further improved the performance of the generated visual stimulus images in terms of subjective visual perception and objective image quality by introducing the visual consistency item into the CNN model during this stage.

## 5. Conclusions

Biomedical signal processing and analysis technology is the core of biomedical informatics research. In recent years, with the rapid development of biomedical-related disciplines represented by medical imaging and brain science, the demand for large-scale, multi-mode biomedical signal processing in this field has increased dramatically, and the method of relying solely on researchers to analyze data manually has been far from meeting the requirements of timeliness. Due to the shortage of model feature expression ability and model capacity, biomedical signal analysis methods based on traditional machine learning methods have become increasingly inadequate in data processing and analysis accuracy. The actual accuracy of the method in the article is above 90% on average. In particular, traditional machine learning methods are difficult to improve in the face of image data with varied visual characteristics, such as mammary gland images, and sequence signals, such as EEG, which are easily affected by the external environment. Aiming at the classification and reconstruction of the two representative biomedical signals, the image of breast mass and the EEG signal, a series of signal analysis methods based on CNN model are proposed in this paper.

In the face of the problem of classification of breast lumps, the existing methods based on traditional manual visual feature representation cannot effectively describe the visual characteristics of breast lumps at different levels, which seriously affects the classification performance of subsequent classifiers on this task. This paper presents a classification method of benign and malignant breast lumps based on CNN feature representation. By analyzing the performance of this method from both subjective and objective aspects, the experimental results show that this method can effectively improve the classification accuracy of breast masses based on mammography images. Traditional methods of EEG signal classification usually only consider the spatial or temporal characteristics of EEG signals and cannot make full use of the abundant spatiotemporal information of EEG signals. In addition, due to the strong randomicity and intra-class diversity of the signals themselves, the traditional manual features are often unable to obtain the high-level consistency information in the same type of EEG signals and the distinguishing features between different types of EEG signals. To solve this problem, an EEG signal classification method based on spatiotemporal fusion CNN is proposed in this paper. The model includes two feature representation networks focusing on temporal and spatial characteristics of EEG signals, and a feature fusion structure combining the two types of feature representations. The two feature representation networks can obtain the high-level features for effective characterization of EEG signals, respectively. The feature fusion structure can further improve the classification accuracy of EEG signals by screening the components related to classification tasks in the two feature representations. We used the proposed method to carry out classification experiments on EEG signal data sets related to working memory, and the experimental results showed that the spatial-temporal fusion CNN model could effectively improve the accuracy of EEG signal classification while maintaining model parameters of a smaller magnitude. In the neural decoding method of visual stimulation based on EEG signals, the characteristics of EEG signals in cognitive space are usually described, and then the classification and reconstruction of visual stimuli are carried out through this feature description. However, there is a certain perceptual bias in the neural response of human brain under external stimulation, which will be further amplified in the process of neural signal acquisition. The above characteristics make the upper limit of the accuracy of visual stimulus decoding restricted by the validity of neural signal characteristics, so it is difficult to continue to improve. At present, with the powerful feature representation ability of deep learning model, the performance of CNN-based visual classification method in vision-related tasks has surpassed the human level. Inspired by this, this paper proposes a visual stimulus reconstruction method based on generation against CNN in order to break through the restriction of the effectiveness of the representation of single neural signal features. The method includes EEG signal classification and visual stimulus generation. In the EEG signal classification stage, the EEG signal classification guided by visual features is realized by returning the EEG signal features to the corresponding visual feature representation. At the stage of visual stimulus generation, the traditional generation versus CNN model was improved by introducing visual consistency preserving items, and the task of visual stimulus reconstruction was completed by visually guided EEG features to generate high-quality visual stimulus images. Finally, the proposed method is verified on the largest EEG signal decoding data set, and the experimental results show that this method can effectively improve the subjective perception and objective evaluation index of the reconstructed visual stimulus.

With the introduction of deep learning methods represented by CNN into the field of biomedical informatics, the problem of insufficient capability of traditional feature representation methods in the face of diversified and large-scale biomedical signals can be solved to a certain extent. However, with the emergence of new interdisciplinary research represented by brain science, how to comprehensively analyze and utilize multi-mode biomedical signals in different application scenarios has become a new challenge in the field of biomedical informatics. Due to the author's lack of ability, there are many mistakes in the experimental part. Due to the difference of the experimental environment, there may be distortions in the data. The author will continue to study hard and do better in the future work.

## Figures and Tables

**Figure 1:** Relationships between biomedical informatics and other disciplines.

**Figure 2:** Directed acyclic graph representation of CNN.

**Figure 3:** Classification accuracy of breast masses by different methods.

**Figure 4:** CNN feature distribution visualization of tumor. (a) The underlying characteristics. (b) Conv5. (c) Fc7.

**Figure 5:** Classification accuracy of EEG signals.

**Figure 6:** Visualized distribution of EEG features in visual guidance. (a) EEG. (b) EEG-Alex. (c) EEG-Res50. (d) EEG-Res101.

**Table 1:** The statistics of common working.

Males			Females		
Prostate	180890	21%	Breast	246660	29%
Lung and bronchus	117920	14%	Lung and bronchus	106470	13%
Colon and rectum	70820	8%	Colon and rectum	63670	8%
Urinary bladder	58950	7%	Uterine corpus	60050	7%
Melanoma of the skin	46870	6%	Thyroid	49350	6%
Non-Hodgkin lymphoma	40170	5%	Non-Hodgkin lymphoma	32410	4%
Kidney and renal pelvis	39650	5%	Melanoma of the skin	29510	3%
Oral cavity and pharynx	34780	4%	Leukemia	26050	3%
Leukemia	34090	4%	Pancreas	25400	3%
Liver and intrahepatic bile duct	28410	3%	Kidney and renal pelvis	23050	3%
All sites	841390	100%	All sites	843820	100%

**Table 2:** *D* main parameters of each layer of network.

The name	Filter size	Filter dimension
Conv1	4	64
BN	—	—
ReLU1	1	—
Conv2	4	128
BN	—	—
ReLU2	1	—
Conv3	4	256
BN	—	—
ReLU3	1	—
Conv4	4	512
BN	—	—
ReLU4	1	—
Fc5	1	1024
BN	—	—
Fc6	1	40

**Table 3:** Comparison with other convolutional neural network models.

Tumor classification method	The storage space (MB)	The number of arguments	Classification accuracy (%)
AlexNet	233	6.1*e* + 07	92
VGGNet	528	1.4*e* + 08	97
Ours	204	5.8*e* + 07	96.7

## Data Availability

Data sharing is not applicable to this article as no new data were created or analyzed in this study.
